# Efficacy of Phase II Remote Home Rehabilitation in Patients with Acute Myocardial Infarction after Percutaneous Coronary Intervention

**DOI:** 10.1155/2022/4634769

**Published:** 2022-06-13

**Authors:** Zhe Li, Zhi Hui, Ye Zheng, Jing Yu, Jun Zhang

**Affiliations:** ^1^Department of Cardiac Rehabilitation, Cangzhou Teaching Hospital of Hebei Medical University, Cangzhou Central Hospital, Cangzhou, Hebei, China; ^2^ICU, Cangzhou Teaching Hospital of Hebei Medical University, Cangzhou Central Hospital, Cangzhou, Hebei, China; ^3^Department of Cardiology, Cangzhou Teaching Hospital of Hebei Medical University, Cangzhou Central Hospital, Cangzhou, Hebei, China

## Abstract

**Objective:**

To assess the efficacy of home-based cardiac rehabilitation and traditional outpatient rehabilitation in stage II after percutaneous coronary intervention (PCI) in patients with acute myocardial infarction (AMI).

**Methods:**

From September 2019 to March 2020, 80 AMI patients in Cangzhou Central Hospital were randomly assigned to one of the two groups: the control group or the observation group, 40 cases in each group. The control group received old-fashioned outpatient rehabilitation treatment, and the study group received long-distance family rehabilitation nursing intervention. The blood pressure, examination results, compliance, satisfaction evaluation, incidence of cardiac events, heart rate, quality of life score, and 6-minute walking test were compared between the two groups.

**Results:**

There were no deaths in both groups. There were significant differences in heart failure, unstable angina pectoris, unplanned readmission rate, walking compliance, and 6-minute walking test at 6 months after discharge (*P* < 0.05). There were substantial variances in left ventricular discharge portion, low-density lipoprotein, medication compliance, satisfaction, and quality of life (*P* < 0.05); there was substantial inconsistency in the 6-minute walking test concerning the two groups afterwards discharge for 3 months (*P* < 0.05).

**Conclusion:**

Home rehabilitation is a new home cardiac rehabilitation model with high efficiency, convenience, and whole process monitoring and barrier-free follow-up management. It can effectively improve the cardiac function, workout patience and worth of life expectancy of victims with AMI, improve their self-management awareness and rehabilitation compliance, reduce the risk of cardiac events, and have a positive impact on the prognosis and rehabilitation of patients with AMI.

## 1. Introduction

Acute myocardial infarction (AMI) is caused as a result of severe and lasting ischemia or necrosis of the corresponding myocardium because of the sharp drooping or interruption of blood supply on the basis of coronary artery dysfunction [1]. AMI is the primary reason of disability and demise in China. At present, the treatment technology of cardiovascular diseases in China has reached the international advanced level, but AMI patients after PCI still face high mortality, cardiovascular disease recurrence rate, and rehospitalization rate, resulting in huge expenditure of medical expenses and patients' confusion and dissatisfaction with medical results. The reasoning behind high mortality is that patients who survived of an earliest acute myocardial infarction (MI) have stroke, high danger of demise, heart failure, arrhythmias, and frequent MI and angina, among other things. Patients (and their families) frequently inquire about their prognosis following MI; hence, prognosis information is essential for patient management.

Cardiac rehabilitation and prevention can fundamentally reverse the simple biomedical model. Cardiac rehabilitation reduces the sudden death rate, recurrence rate, and readmission rate of cardiovascular disease through the combination of five core prescriptions (prescription, exercise prescription, nutrition prescription, psychological prescription, risk factor management, and smoking cessation prescription). Cardiac rehabilitation can be divided into three stages: stage I, hospitalization rehabilitation, 4–7 days after onset; II stage, outpatient rehabilitation, 7 days to 3–6 months after onset; and the third stage, family rehabilitation, from 6 months after onset to the whole life process [2]. The traditional second-stage cardiac rehabilitation exercise therapy begins within 1–3 weeks after discharge and lasts for up to 36 weeks when clinical conditions permit. The frequency is generally 3 days a week. Usually, clinical monitoring is needed at this stage to ensure the safety of exercise therapy. The exercise rehabilitation of patients with AMI in China is still in its infancy, lack of scientific and effective monitoring methods. Considering the economic cost, traffic obstacles, and place of residence, most patients prefer home cardiac rehabilitation after discharge [3]. Recent studies have shown that home cardiac rehabilitation can improve patients' prognosis as well as traditional cardiac rehabilitation and greatly improve patients' quality of life, save medical costs, and improve patients' compliance. A recent foreign study found that smartphone-based cardiac rehabilitation software can guide the overall course and quality of exercise for patients with heart disease [4].

Therefore, the proposed study on victims with acute myocardial infarction PCI postoperative stage II remote home rehabilitation, compared with old style casualty rehabilitation efficacy [5], hope by the aid of remote ECG detection technology [6], real-time, and incessant intensive caring of the patient's health auxiliary PCI postoperative patients having acute myocardial infarction, the guidance of doctors treatment outside the hospital rehabilitation treatment and health management for a long time to make the rehabilitation management and follow-up of AMI patients precise and standardized [7], so as to improve patient compliance, further improve the continuity of AMI patients' diagnosis and treatment in and out of the hospital, reduce patients' rehospitalization rate and mortality, and improve the worth of life.

## 2. Methods

### 2.1. Participants

Eighty patients having acute myocardial infarction who received emergency PCI in Cangzhou Central Hospital in the period of September 2019 to March 2020 were nominated for the examination as objects. The parallel randomized control method was used in the proposed study, and selected patients were arbitrarily allotted to one of two groups: observation or control, considering 40 cases for each group. In the observation group, there were 27 males and 13 females, (55.4 ± 8.9) years old, while in the control group, 25 males and 15 females, (55.6 ± 8.3) years old. There was no significant difference in general data between the two groups (*P* > 0.05). Participants in randomized controlled trials are randomly allocated to either the treatment or control arms. The practice of arbitrarily allocating sample members to treatment or control arms is referred to as randomization. To randomly select, a variety of tools can be utilized (closed envelopes, computer-generated sequences, and random numbers). The two factors of randomization are the creation of a random pattern and the implementation of such a random pattern, ideally in a way that leaves participants unaware of the sequence (allocation concealment). The danger of systematic error or prejudice is eliminated by randomization. The most important benefit of an RCT is that it accounts for both predictable and unpredictable confounding variables, which can result in errors.

Inclusion criteria were as follows: met the diagnostic criteria for acute myocardial infarction (4th edition global definition of myocardial infarction) [8]; emergency PCI was performed for the first time, and all the enrolled patients received emergency PCI through the radial artery of the upper limb as the puncture approach; the risk stratification of coronary heart disease was low to medium risk, cardiac function Killip grade was I-II, and cardiac ejection fraction >50%; age from 30 to 70; good understanding and communication skills; and volunteer to participate in the proposed study.

Exclusion criteria were as follows: the history of myocardial infarction; there are serious complications, such as cardiogenic shock, severe arrhythmia, severe congestive heart failure, hypotension, obvious persistent or episodic chest pain, and mechanical complications; a history of mental disorders; serious other diseases, such as serious cerebrovascular disease sequelae, mobility inconvenience and physical disability and other factors affecting sports, severe anemia, and serious chronic lung diseases.

### 2.2. Study Protocol

Exercise prescriptions were formulated as stated by the strategies of the American College of Sports Medicine [9], and the walking program for patients with standardized AMI after discharge was set. The observation group received standardized health education, distributed walking program after discharge, medication list, and precautions, and were documented by nurses. The research group set up a medical rehabilitation team, which was divided into 6 groups according to the doctor in charge and set up 6 WeChat groups. Each group had 1 doctor and 1 nurse tracking the implementation process of the exercise program. The patients were taught by the nurses about the Borg grading of self-evaluation of fatigue (Borg grading), and the Borg grading remained at 11–14 after exercise [10]. The Borg scale is a tool used to assess a person's feeling of effort, exertion, dyspnea, and exhaustion when performing physical tasks. Patients were taught to monitor their heart rate using checkup app or exercise bracelet, and the maximum heart rate was required to be resting plus 20–30 times/min after exercise [10]. Nurses track patients' medication and exercise completion through “daily list” supervision and collect and record patients' heart rate, Borg grade, and other discomfort after exercise. Physicians are responsible for answering patients' questions and adjusting medication regimen and exercise intensity. A telephone follow-up group was set up for the control group, including 2 nurses for telephone follow-up. The patients were followed up by telephone once a week, focusing on asking them whether they took medicine on time, exercised, and had any discomfort and recording them. The patients' problems were fed back to the doctor by the nurse for timely treatment. The control group received traditional outpatient rehabilitation. In this study, all patients were followed up, and there was only one patient who had a second myocardial infarction during the follow-up period.

### 2.3. Termination Motion Indication

Chest tightness, chest pain, and shortness of breath appear after exercise. The heart rate after activity was lower than 50 beats/min or more than 130 beats/min. Postactivity Brog rating was >15.

### 2.4. The Index of Evaluation

Walking frequency ≥50 times is considered as compliance standard [11]. Those who did not follow the doctor's advice to take medicine for more than 10 times were considered as substandard medication compliance. If the frequency of return visit is less than 2 times, the compliance of return visit is not up to standard.

### 2.5. Observation Index

The nurses collected and sorted out the patients' heart rate, blood pressure, laboratory results, compliance, satisfaction assessment, incidence of cardiac events, quality of life score, and 6-minute walking test.

### 2.6. Statistical Analysis

The statistical software SPSS 17.0 was used to analyze the data. The statistical data were expressed as percentage (%), and the *χ*^2^ test was used. *P* < 0.05 was considered as statistically major difference.

The chi-square 2 statistic measures the difference between the observed and predicted probabilities of the consequences of a series of actions or variables. The chi-square test is a useful tool for determining category differences, especially those that are only nominal. The sample size, the degree of freedom, and the amount of the disparity in actual and recorded values all have an impact on the value of *χ*^2^. The *χ*^2^ test could be used to evaluate if two variables are highly correlated or not.

## 3. Results

### 3.1. Comparison of Compliance Evaluation Results

The difference of walking and medication compliance was statistically significant (*P* < 0.05) (See Tables 1–5 for details).

The difference of unplanned readmission rate was statistically significant (*P* < 0.01); there were significant differences in LDL, satisfaction, and left ventricular ejection fraction (*P* < 0.05).

Most of your body's cholesterol is made up of LDL (low-density lipoprotein), also known as “bad” cholesterol. LDL cholesterol levels that are too high put you at risk of heart disease and stroke.

To compute LDL, the following given formulation is used:

(1) $$\begin{array}{c} \text{LDL}=\text{Total cholestrol }\left(\frac{\text{triglyceride}}{5}\right)-\text{HDL}. \end{array}$$

There was major change in the occurrence of unstable angina pectoris and congestive heart failure (*P* < 0.01). There was no substantial change in the occurrence and mortality of reinfection (*P* > 0.05).

There was no statistically substantial transformation between the 6-minute walking test at releasing and one month later (*P* > 0.05). 3 months after discharge, the difference was statistically significant (*P* 0.05). The variance was statistically substantial 6 months after discharge (*P* < 0.01).

There was significant difference in the scores of life quality between the two groups at 6 months after discharge (*P* < 0.05).

## 4. Discussion

The remote home rehabilitation mode of “Internet+ integrated medical care rehabilitation team” was applied to form a comprehensive, quantitative, individual, and sustainable new mode of home exercise rehabilitation, which improved the participation and safety of cardiac rehabilitation for AMI patients [12]. The proposed study showed that at 6 months after discharge, the incidence of congestive heart failure, unstable angina pectoris, the study group's unplanned readmission rate, and aberrant left ventricular ejection fraction were pointedly lesser (*P* 0.05) than the control groups, whereas the 6-minute walking test and quality of life were significantly greater (*P* 0.05). The rates of reinfection and mortality in the two groups were not significantly different. Home rehabilitation may help AMI patients improve their heart function, activity tolerance, and quality of life, but not increase the incidence of cardiac events and mortality, so it is safe and feasible for patients.

AMI guidelines of the European Cardiology Society in 2012 pointed out that walking is the best way for stage II rehabilitation of AMI patients [13]. Since each patient has completely different cardiac function and exercise tolerance, it is particularly important to define walking speed and distance, control exercise intensity, and select a universal walking program. In the absence of specialized rehabilitation institutions and teams, safety is the primary consideration for stage II cardiac rehabilitation in patients with AMI [14]. In [15], the foreign mature walking program was used for preexperiment, and the standardized walking program for AMI patients for 6 months after discharge was revised. The activity volume increased every 2 weeks, ensuring the safety and scientific nature of home exercise rehabilitation.

According to some researchers, cardiac rehabilitation must be done through exercise under medical observation [16]. In the absence of specialized rehabilitation institutions, the checkup app or exercise bracelet can help medical staff monitor heart rate in real time and complete continuous medical observation of home rehabilitation. However, the continuous heart rate monitoring of checkup app or exercise bracelet cannot completely replace the evaluation and analysis of medical staff. To control the risk factors of home exercise rehabilitation for AMI patients, it is necessary to combine the accessible follow-up management of the WeChat group of the integrated medical rehabilitation team, dynamic evaluation of integrated medical care, online follow-up at any time, real-time supervision, and feedback. Multiple guarantee for the safety of cardiac exercise rehabilitation at home. WeChat daily checklist follow-up management, in the mode of “compulsion to promote consciousness,” enables patients to participate in rehabilitation from passive to active, from supervision to consciousness, and improves compliance and rehabilitation confidence.

Six months after discharge, the walking compliance of patients in the control group was only 50% (20/40) and that of patients in the study group was about 95% (38/40), which was similar to foreign studies [17]. Two groups are in the rehabilitation period; all experience the excitement period, quiet period, the relief phase stage, restart, recession, achievement six stages, how to break through the relief phase, decline phase which is the focus in the study of cardiac rehabilitation exercise that occupy the home, best can establish in patients with cardiac rehabilitation club, by the medical staff involved in tracking guidance all the way, give play to the role of compliance in patients with good incentive, and mobilize family members or caregivers to participate in the guidance, help patients build confidence in rehabilitation, establish personal rehabilitation movement energy cycle, adhere to rehabilitation and self-management, and truly improve the quality of life [18, 19].

In this respect, we suggest a procedure for implementing a statistical approach to questionnaire validation that incorporates exploratory factor analysis and reliability analysis. The research focuses on the psychometric examination of data from a survey.

The home cardiac rehabilitation mode effectively ensures the safety and scientific nature of stage II home rehabilitation for AMI patients, improves patient compliance and quality of life, and is worthy of promotion through the standardized walking program, real-time monitoring of heart rate by APP or exercise bracelet, and barrier-free follow-up management on WeChat platform of medical rehabilitation team. The limitation of the projected study is that only exercise and medication intervention were carried out. With the development of information technology and cloud technology, more rehabilitation procedures and simple and effective monitoring equipment should be developed in the future, and behavioral intervention should be included in the stage II cardiac rehabilitation of AMI patients, so as to make cardiac rehabilitation more humanized, individual, convenient, and systematic.

## Figures and Tables

**Table 1:** Comparison of compliance evaluation between two groups of patients with acute myocardial infarction 6 months after discharge (*n*).

Index	Control group (*n* = 40)	Observation group (*n* = 40)	*P*
Medication compliance	28	37	<0.05
Walking compliance	20	38	<0.05
Compliance of return visit	37	40	>0.05

**Table 2:** Comparison of cardiac function, satisfaction, and low-density lipoprotein/unplanned readmission rate between the two groups of patients with acute myocardial infarction 6 months after discharge (*n*).

Index	Control group (*n* = 40)	Observation group (*n* = 40)	*P*
LVEF <50%	8	3	<0.05
Unplanned readmission rate	7	1	<0.01
Satisfaction (%)	77.50	92.50	<0.05
LDL (mmol/L)	26.78 ± 3.65	23.17 ± 2.58	<0.05

**Table 3:** Comparison of the occurrence of antagonistic cardiac proceedings 6 months subsequently discharge concerning two groups of acute myocardial infarction patients (*n*).

Index	Control group (*n* = 40)	Observation group (*n* = 40)	*P*
Second myocardial infarction	1	0	>0.05
Unstable angina	8	2	<0.05
Congestive heart failure	7	1	<0.05
Case fatality rate	0	0	>0.05

**Table 4:** Comparison of the 6-minute walking test between two groups of patients with acute myocardial infarction (*m*).

Time	Control group (*n* = 40)	Observation group (*n* = 40)	*P*
1 month	278.68 ± 30.28	282.96 ± 30.77	>0.05
3 months	309.74 ± 34.89	332.85 ± 35.88	<0.05
6 months	346.72 ± 42.96	421.75 ± 45.96	<0.05

**Table 5:** Comparison of the scores of life quality between two groups of patients with acute myocardial infarction (score).

Time	Control group (*n* = 40)	Observation group (*n* = 40)	*P*
At discharge	63.85 ± 7.26	64.59 ± 6.78	>0.05
6 months after discharge	77.35 ± 9.21	89.46 ± 9.33	<0.05

## Data Availability

The datasets used and analyzed during the current study are available from the corresponding author upon request.
